# Recognition of Unknown Entities in Specific Financial Field Based on ERNIE-Doc-BiLSTM-CRF

**DOI:** 10.1155/2022/3139898

**Published:** 2022-05-14

**Authors:** Li Xin, Hao Xiaoyan

**Affiliations:** College of Information and Computer, Taiyuan University of Technology, Taiyuan, Shanxi 030000, China

## Abstract

The Internet is rich in information related to the financial field. The financial entity information text containing new internet vocabulary has a certain impact on the results of existing recognition algorithms. How to solve the problems of new vocabulary and polysemy is a problem to be solved in the current field. This paper proposes an ERNIE-Doc-BiLSTM-CRF named entity recognition model based on the pretrained language model. Compared with the traditional model, the ERNIE-Doc pretrained language model constructs a unique word vector from the word vector and combines the location coding, which solves polysemy problem well. The intensive skimming mechanism realizes the long text processing well and captures the context information effectively. The experimental results show that the accuracy of this model is 86.72%, the recall rate is 83.39%, and the F1 value is 85.02%, which is 13.36% higher than other models; the recall rate is increased by 13.05%, and the F1 value is increased by 13.21%.

## 1. Introduction

Named entity recognition (NER) refers to the recognition of text fragments belonging to predefined categories from free text. NER task was formally proposed for the first time at the sixth message understanding conference. At that time, only some general entity categories were defined, such as location, organization, and person [1]. At present, the task of named entity recognition has penetrated into various vertical fields, such as medical treatment, finance, and so on. The named entity recognition algorithm was first applied to NER by Sekine et al. [2] in 1998, and Borthwick et al. [3] applied the maximum entropy model to NER at the same time. This was followed by bootstrapping learning by Collins and Singer [4] in 1999 using a small prelabeled data set (seed data). The relatively mainstream conditional random field model was first applied to NER in 2003 by McCallum and Li et al. [5]. Because the conditional random field model is easy to implement and has certain performance, it is very popular among NLP researchers and is widely used in various types of entity recognition such as person names, place names, time, currency, and organizations. It is one of the most widely used and one of the most successful methods. In recent years, the development of deep learning has progressed steadily, and the use of deep learning in named entity recognition tasks has also become a new trend. Among them, the most commonly used is a recurrent neural network (RNN) and its variants that can capture sequence information, such as long short-term memory (LSTM) network and its improved bidirectional long- and short-term memory (BiLSTM) network. Reference [6] proposed a self-trained BiLSTM-CRF model for Chinese NER tasks. There are also researchers using convolutional neural network (CNN) to identify entities, such as Zhu et al. [7] using CNN to encode Chinese characters. Wang Jie et al. [8–10] adopted the GRU computing unit in the meeting name task and proposed a GRU-based named entity recognition method.

Unknown entity recognition in specific financial fields refers to extracting unknown financial entities from unlabeled and unstructured Internet texts. In recent years, with the development of the Internet, traditional offline facade loans and loan advertisements all over the place are gradually being transferred online, resulting in a large number of internet texts containing advertising information. Extracting these financial entity information from internet texts can help relevant institutions better build monitoring systems. However, in order to avoid supervision, these texts use traditional Chinese, symbolic phrases, pinyin, and so on, which has caused great difficulties in extracting financial entity information. Manually extracting these financial entities from massive internet texts will consume a lot of manpower and time, and it is particularly important to use an efficient and accurate algorithm to solve this problem as shown in Figure 1.

To this end, a large number of scholars have begun to try to obtain prior semantic knowledge from a large amount of unlabeled text to enhance semantic representation and apply it to various NLP tasks such as named entity recognition. Google Brain proposes transformer-based pretraining models, such as BERT (bidirectional encoder representations from transformers). BERT obtains prior semantic knowledge from unlabeled text through two pretraining tasks, masked language model (MLM), and next sentence prediction (NSP), while fine-tuning downstream task parameters to apply the enhanced semantic representation containing these knowledge to downstream natural language processing tasks, such as recognizing named entities in Chinese electronic medical records [11], with the help of pretrained language models, good results can be achieved. However, the BERT model has inherent deficiencies when dealing with Chinese tasks. It adopts random strategies for masking training for word granularity and does not make full use of lexical data and grammatical structures. The word handles random masks separately, ignoring the lexical information of “Apple phone,” so the universality of the model is affected, and it is difficult to obtain a good semantic representation for emerging mobile phone brands. At the same time, BERT is limited by the maximum input length of the model. When encountering long sentences, it has to be segmented, which is not conducive to the capture of contextual information.

Aiming at the above problems, this paper proposes an unknown entity recognition model in a specific financial domain based on ERNIE-Doc-BiLSTM-CRF (EDBC). Compared with the traditional combination of Word2Vec-BiLSTM-CRF and different downstream models, the experimental results show that this model can effectively improve the recognition effect of unknown entities in specific financial fields.

## 2. EDBC Algorithm Model

ERNIE-Doc-BiLSTM-CRF is an unknown financial entity recognition model proposed in this paper. Its main mechanism first obtains the semantic representation of each word and, then for each word, combined with position encoding, according to certain rules, takes the corresponding position. The hidden layer parameters are feature-fused to obtain a unique semantic representation of each word with contextual information. At the same time, an improved self-attention mechanism is used to calculate the weight of each word in the input text synchronously, to learn the dependencies of each word in the sentence, and to obtain the internal structure of the sentence. The closely related bidirectional LSTM network double-models the multidimensional vectors containing the internal representation of the sentence and splices it to obtain the updated semantic representation of the sentence. Finally, after being processed by the CRF decoding module, the label sequence is further optimized according to the preset rules to obtain the optimal solution. The data collection of this study mainly comes from Baidu Encyclopedia, web pages, manual texts, and other massive databases with uniquely identified word vectors. Since each word is a uniquely identified word vector, the relevant data information is valid. The bidirectional LSTM network further extracts the contextual information of the text and finally uses a conditional random field (CRF) to limit the sequence relationship between labels. The EDBA model includes an input layer, a pretrained language model layer, a BiLSTM layer, and a CRF layer. The model structure is shown in Figure 2.

### 2.1. ERNIE-Doc Module

With the exploration of a large number of scholars, it has become a consensus that the semantic representation of downstream tasks using pretraining models (PTMs) trained on very large corpora in advance has good results, saving the time of training models for downstream tasks. PTMs have been developed for two generations so far. Among them, the first-generation PTMs represented by the well-known Word2Vec and GloVe models have learned the embedding of a single word well, but there is no effective solution for the context relationship, such as sentence relationship, syntactic structure, polysemy, and so on. The second-generation PTMs are designed to solve the intersentence isolation phenomenon in the first-generation PTMs. For example, the ELMo model using bidirectional LSTM can capture contextual information well, but there is only one layer of bidirectional LSTM network; OpenAI GPT uses a unidirectional LSTM network. The transformer structure can only capture context information in one direction; the full name of ERNIE-Doc is Enhanced Language Representation with Informative Entities-Doc, and the structure is shown in Figure 3.

The core part of ERNIE-Doc is the multilayer transformer structure, which mainly includes position encoding and self-attention mechanism. Compared with the traditional recurrent neural network, the ERNIE-Doc model solves the problems of distraction and long training time in the face of long text by using a multilayer self-attention mechanism. Among them, self-attention is one of the attention mechanisms and an important part of the transformer [12].

The core part of ERNIE-Doc is the multilayer transformer structure, which mainly includes two parts: position encoding and self-attention. Among them, compared with the traditional recurrent neural network, the ERNIE-Doc model adopts a multilayer self-attention mechanism (self-attention), which well solves the problems of distraction and long training time in the face of long texts. Among them, self-attention is one of the attention mechanisms and an important part of the transformer. Its operation mechanism is mainly to use multihead self-attention to connect the encoder to the decoder and multiply the word vector after word embedding with the *W*_*q*_, *W*_*k*_, and *W*_*v*_ weight matrix to obtain the query vector (*Q*), key vector (*K*), and value vector (*V*); then the importance of each word multiplied by the *Q* vector and the *K* vector is softmax normalized; and finally, this value is multiplied by *V* to obtain the processed word vector. The correlation between words is obtained by calculating the attention between each word in the sentence, which further captures the structure of the sentence. The attention calculation formula, such as (1), is a dimension of *Q* and *K*, and $\sqrt{d_{k}}$ is introduced as a penalty factor to ensure that the inner product of *Q* and *K* is within a reasonable range.

(1) $$\begin{array}{c} \text{Attention }\left(Q,K,V\right)=\text{softmax}\left(\frac{{\text{QK}}^{T}}{\sqrt{d_{k}}}\right)V\text{.} \end{array}$$

Improvements have been made here when calculating attention. The calculation time and memory usage of self-attention are square. If the sequence length becomes 2 times the original, the memory usage is 4 times the original, and the computing time is also 4 times the original. Therefore, sparse self-attention is adopted, and the attentions with the relative distances not exceeding *k* ± 3, 2*k* ± 3, 3*k* ± 3… are set to 0, so that when calculating attention, it has the characteristics of local close correlation and long-distance sparse correlation.

Since the calculation process of attention does not depend on the order between words in the sentence, but the information is mined by calculating the similarity between words, we can carry out multiple sets of attention training at the same time, so the speed of training is obtained. While greatly improving, it also avoids the problem of information loss caused by too long sequences. But, because of this, we need to mark the sequence of each word in the sentence through Position Embedding. At the time of word embedding calculation at time *t*, a position vector closely related to time *t* is introduced, and the two are spliced together as the input of the model. For the problem that the same word appears multiple times in a sentence, since the time *t* of each word appears is different, although the vector encoding of the same word is the same, the final vector is also unique.

By repeatedly inputting long text into the model twice, ERNIE-Doc learns and stores the semantic information of the whole text in the rough reading stage, and explicitly integrates the semantic information of the whole text for each text segment in the intensive reading stage, thereby realizing bidirectional modeling and avoiding the need for the problem of context fragmentation. The calculation in the rough reading stage is shown in (2), and the calculation in the intensive reading stage is shown in (3):

(2) $$\begin{array}{c} \hat{H}=\left[{\hat{H}}_{1:T}^{1}\circ {\hat{H}}_{1:T}^{2}\cdots \circ {\hat{H}}_{1:T}^{N}\right], \end{array}$$

(3) $$\begin{array}{c} {\tilde{h}}_{\Gamma +1}^{n-1}=\left[\text{SG}\left(\hat{H}\circ h_{\Gamma }^{n-1}\right)\circ h_{\Gamma +1}^{n-1}\right], \end{array}$$

where $\hat{H}\in R^{\left(L*T*N\right)\times d}$ represents the hidden state of the text *T* in the skimming phase, *L* represents the length of each segment, *N* represents the total number of layers, SG(·) represents the gradient descent algorithm, and ${\hat{H}}_{1:T}^{i}=\left[{\hat{h}}_{1}^{i}\circ {\hat{h}}_{2}^{i}\cdots \circ {\hat{h}}_{T}^{i}\right]$ represents the *i*-th hidden layer connection in the skimming phase. In this way, ${\tilde{h}}_{\Gamma +1}^{n-1}$ is guaranteed to capture bidirectional contextual information for the entire document.

In addition, the recurrent way of the recurrence memory structure in traditional long text models (Transformer-XL, etc.) limits the effective modeling length of the model. ERNIE-Doc improves it into a same-layer loop, obtains the output of the previous moment and the next, and supports a larger length so that the model retains the semantic information of the upper layer and has the modeling ability of superlong text. Finally, ERNIE-Doc better models the overall information of the text by letting the model learn the sequential relationship between text paragraphs at the text level.

### 2.2. BiLSTM Module

Recurrent neural network (RNN) is a type of neural network for processing sequence data [13]. Due to the natural advantages of this kind of network model structure in the field of natural language processing, it has been widely used once it was proposed. For named entity recognition tasks, the forward and backward information of sentences will have a huge impact on text understanding, and the traditional one-way recurrent neural network can only capture one-way historical information. Therefore, bidirectional RNN (BRNN) was proposed by Graves et al. [14] in 2013, and the improved model was successfully applied to the task of named entity recognition and achieved good results beyond the previous ones. The bidirectional long short-term memory (LSTM) network used in this paper is obtained by adjusting the structure of the traditional RNN and is a variant of the LSTM network proposed by Hochreiter and Schmidhuber in 1997 [15], which effectively solves the problem of gradient disappearance and gradient explosion in the face of long texts. Due to the addition of the forgetting gate, compared with the traditional RNN, the performance of LSTM in longer sequences is significantly improved.

In the following time, Graves further proposed an improved BiLSTM model, which can make good use of the forward and backward information of sentences and improve the ability of the model to use context information. As shown in Figure 2, the output of the aforementioned ERNIE-Doc module will be used as the module's output.

The basic unit calculation method of LSTM is shown in the following formulas:

(4) $$\begin{array}{c} z=\tanh\left(W\frac{x^{t}}{h^{t-1}}\right),\\ z^{i}=\sigma \left(W^{i}\frac{x^{t}}{h^{t-1}}\right),\\ z^{f}=\sigma \left(W^{f}\frac{x^{t}}{h^{t-1}}\right),\\ z^{o}=\sigma \left(W^{o}\frac{x^{t}}{h^{t-1}}\right). \end{array}$$

Among them, the three state calculation methods are shown in the following formulas:

(5) $$\begin{array}{c} c^{t}=z^{f}⊙c^{t-1}+z^{i}⊙z,\\ h^{t}=z^{o}⊙\;\tanh\left(c^{t}\right),\\ y^{t}=\sigma \left(W^{\prime }h^{t}\right). \end{array}$$

Among them, *z*^*f*^, *z*^*i*^, and *z*^*o*^ are three gated states, which are obtained by multiplying the splicing vector by the weight matrix and then converting it into a value between 0 and 1 through the sigmoid activation function. Instead, the result is converted into a value between –1 and 1 through a tanh activation function; *W*, *W*^*i*^, *W*^*f*^, and *W*^*o*^ are all trainable parameters; 88 is the memory state in the LSTM unit; and *c*^*t*^ is the LSTM unit. The hidden layer state of the previous layer, *h*^*t*−1^, is the output of the current state, and *y*^*t*^, *σ*, and tanh are activation functions.

### 2.3. Decoding Module

In the named entity recognition task, adjacent labels often have dependencies. Although the BiLSTM module fully considers the contextual semantic information, it lacks restrictions on the order relationship between labels. For example, the common rule is that any sentence always starts with the label “B” or “O,” the label “I” must appear after the label “B” and so on.

Conditional random field (CRF) is the most widely used serialization labeling algorithm, proposed by Lafferty et al. in 2001 [16], and the Viterbi algorithm is usually used for training and decoding linear conditional random fields [17]. The CRF decoding module is introduced, and some constraints can be added to the predicted labels to constrain the validity of the label sequence.

Specifically, if for the specified sequence *X*(*x*_1_, *x*_2_,…*x*_*n*_), the corresponding label *Y*(*y*_1_, *y*_2_,…*y*_*n*_) satisfies the condition shown by

(6) $$\begin{array}{c} P\left(Y_{i}|X,Y_{1},\ldots ,Y_{i-1},Y_{i+1},\ldots Y_{n}\right)=P\left(Y_{i}|X,Y_{i-1},Y_{i+1}\right). \end{array}$$

Let *P* (*N*, *K*) be the weight matrix output by the decoding module and obtain the evaluation score *S* (*x*, *y*), as shown in the following equation:

(7) $$\begin{array}{c} S\left(x,y\right)=\sum_{i=0}^{n}A_{y_{i},y_{i+1}}+\sum_{i=1}^{n}P_{i,y_{i}}, \end{array}$$

where *A* is the transition matrix, P_*i*,y*i*_ represents the score of the yi-th label of the character, *k* is the total number of labels, and *n* is the sequence length.

Finally, use softmax to get the normalized probability, as shown in the following equation:

(8) $$\begin{array}{c} P\left(y|x\right)=\frac{\exp\left(\text{score}\left(x,y\right)\right)}{\sum y{}^{\prime }\;\exp\left(\text{score}\left(x,y{}^{\prime }\right)\right)}. \end{array}$$

The probability of the label sequence *Y* is calculated by (8), and the set with the largest probability is selected from it, which is the final label sequence.

## 3. Experiments and Analysis

The data set used in this paper is composed of nearly 10 million words of text provided by the national Internet Emergency Response Center, mainly from the microblog posts, microblog comments, current affairs news, Post Bar Forum, and so on captured by the crawler. In practical application, it is found that there are some label errors in the data set, so some corrections are made. Specifically, when selecting the data set, the corresponding text length distribution is mainly long text; nearly 70% of the text length is more than 500 words; the shortest text is composed of 7 words; the longest text is composed of 37,691 words, and the average length of the whole text is 1,425 words. The training set, verification set, and test set are set according to the proportion of 8:1:1 to ensure the effectiveness of the data set as a whole.

### 3.1. Data Labeling Method and Evaluation Metrics

The data are marked with the BIO three-segment notation method: for each entity, its first word is marked as B– (entity name); B means that the word is at the beginning of an entity (begin); and subsequent marks are I– (entity name), for words that have nothing to do with the current word, it is directly marked as O, and we use O to represent outside. Since the BIO tagging method supports word-by-word tagging, there is no need to presegment the text before the tagging, which avoids the impact of errors caused by word segmentation. Therefore, compared with the BIOES tagging method, this paper chooses the BIO tagging method to mark the data.

For named entity recognition algorithms, three indicators are usually used for evaluation: precision (*P*), recall (*R*), and *F* value, which are defined as the number of correct entities identified by the model, the number of irrelevant entities identified by the model, and the model. The number of related entities that were not detected. The specific formula is shown in the following equations:

(9) $$\begin{array}{c} P=\frac{T_{p}}{T_{p}+F_{p}}\times 100\%, \end{array}$$

(10) $$\begin{array}{c} R=\frac{T_{p}}{T_{p}+F_{n}}\times 100\%, \end{array}$$

(11) $$\begin{array}{c} F_{1}=\frac{2P\times R}{P+R}\times 100\%. \end{array}$$

### 3.2. Experimental Environment

The environment used in all experiments is shown in Table 1.

### 3.3. Data Preprocessing

According to the characteristics of the data set, such as the text contains special symbols such as expressions, various symbols and labels that are not related to the text and so on and methods such as string substitution, regular expression filtering, and replacing noise are adopted to clean the data set. At the same time, BOI encoding is performed on the training set data.

### 3.4. Experimental Setup

The hyperparameters used in this article were found through trial and error.  Table 2 lists some of the hyperparameters used in this paper. During training, in order to find the optimal parameters, multiple rounds of iterations were carried out, and it was finally found that the fifteenth time was the best. In addition, in order to prevent overfitting, drop rate is set to 0.5 in the LSTM layer, and the activation function adopts ReLU to speed up the training speed and further prevent overfitting; the optimizer is Adam; in addition, the gradient clipping technology is used, and the clip is 0.5; set the parameter to 64 in the attention layer.

### 3.5. Experimental Results and Analysis

Throughout the experiment, multiple iterations were performed, and the data of each iteration was compared, as shown in Figure 4. In the graph, the horizontal axis is the number of iterations, and the vertical axis is the percentage. If the number of iterations is too small, it will lead to underfitting, and if the number of iterations is too large, it will lead to overfitting. After experiments, it is found that the data is the best when the number of iterations is 15. At this time, the precision rate, recall rate, and F1 value reach 86.72%, 83.39%, and 85.02%, respectively. When the number of iterations in the early stage is too small, the precision rate, recall rate, and F1 values did not reach the ideal value. When the number of iterations reached 15, the model gradually fitted and became stable at the same time, so the final number of iterations was selected as 15.

In order to reduce the influence of randomness on the results as much as possible, fivefold cross-validation is carried out for the models used in this module. The calculation method is shown in (12), where MSE_*i*_ refers to the mean square error of each result. In the experiment, the value of *k* is 5, and finally, each MSE_*i*_ is averaged to get the final MSE result.

(12) $$\begin{array}{c} {\mathrm{CV}}_{\left(k\right)}=\frac{1}{k}\sum_{i=1}^{k}{\mathrm{MSE}}_{i}. \end{array}$$

In the experiment, the EDBA model and its improved model proposed in this paper are compared with the representative Word2Vec BiLSTM CRF in the field of NER, the famous BERT model in this field, and a series of variants. The experimental results are shown in Table 3.

The overall comparison is shown in Table 3:

In the experiment, the EDBA model proposed in this paper and its improved model are compared with the representative Word2Vec-BiLSTM-CRF in the NER field, the well-known BERT model in the field [18], and a series of variants thereof. The experimental results are shown in Table 3.

It can be seen from Table 3 that since the BERT and EDBC models are based on word embeddings, they have more advantages in capturing the semantic information of the text context. At the same time, the Word2Vec algorithm encodes the same word in exactly the same way, ignoring the possibility that the same word appears in different positions. The semantic change occurs. For example, “The company did not take study documents seriously because everyone was busy with other things when they were asked for.” “Learning documents” appears twice in the sentence, but the meaning is completely different. Therefore, all evaluation indicators have been significantly improved. Compared with the BERT-CRF model, the excellent information extraction capability of the BiLSTM network has been replaced by the bidirectional transformer structure within the BERT model itself. Therefore, the new bidirectional LSTM module in the BERT-BiLSTM-CRF model does not have the result. The experimental results show that the training time is reduced to a certain extent and the recognition effect is not greatly compromised, so it can be used according to actual needs to make a selection. Compared with the BERT-BiLSTM-CRF model, the EDBC model proposed in this paper has a certain improvement in various evaluation indicators. The experimental results show that the accuracy rate of this model is 86.72%, the recall rate is 83.39%, and the F1 value is 85.02% respectively, which is 13.36% higher than that of other models. The recall rate increased by 13.05%; F1 value increased by 13.21%.

## 4. Summary and Outlook

The financial entity recognition model is based on the EDBC word embedding model; the representation will be based on the left and right contexts in all layers and at the same time solve the problem of insufficient reading ability of long texts, so it can capture context information well, compared to traditional models and BERT. The experimental results show that the accuracy of this model is 86.72%, the recall rate is 83.39%, and the F1 value is 85.02%, respectively. The model has a certain improvement in precision, recall, and F1 value.

Benefiting from the domestic environment, the development of my country's financial technology is far ahead of the world average, but it is worth noting that the rapid development of financial technology is diluting the boundaries of traditional financial business, preventing and resolving systemic financial risks, and preventing the transmission of financial risks from breaking through the limitations of time and space. In the face of new challenges, the establishment of the financial entity identification scheme will greatly improve the efficiency of financial information acquisition and then better provide information support for relevant institutions and individuals in the financial field.

## Figures and Tables

**Figure 1:** Identifying unknown financial entities from internet text.

**Figure 2:** Model network structure.

**Figure 3:** Network structure of ERNIE-Doc.

**Figure 4:** Results of different iterations.

**Table 1:** Experimental environment.

Operating system	Windows 10
CPU	Intel Core^TM^ i7-10700F CPU@2.9∗8
GPU	Nvidia RTX 3060 (12 GB)
Python	3.6.5
TensorFlow	1.15
RAM	24 GB

**Table 2:** Hyperparameter used.

Hyperparameters	Numerical value
Epoch	15
Batch size	4
Heads	12
Hidden layer dimension (LSTM)	768
Learning rate	5e-6

**Table 3:** Comparison of results of different models.

Model	Accuracy (%)	Recall rate (%)	F1 value (%)
Word2Vec-BiLSTM-CRF	73.36	70.34	71.81
BERT-CRF	81.72	80.64	81.17
BERT-GRU-CRF	83.23	80.47	81.82
BERT-BiLSTM-CRF	85.49	82.17	83.79
ERNIE-Doc-GRU-CRF	85.91	82.74	84.29
ERNIE-Doc-BiLSTM-CRF	86.72	83.39	85.02
ERNIE-Doc-BiLSTM-CRF∗	86.35	83.09	84.68

## Data Availability

The data set can be accessed upon request.
